This article has been retracted.

# An Evaluation Model of Agricultural Entrepreneurial Ecological Environment Quality Oriented to Public Health Topic Using the Optimized Neural Network Algorithm

**DOI:** 10.1155/2022/8735069

**Published:** 2022-09-16

**Authors:** Xiangmin Meng, Jie Zhang, Guoyan Ren

**Affiliations:** ^1^College of Economics and Management, Nanjing University of Aeronautics and Astronautics, Nanjing, Jiangsu 211100, China; ^2^Business School, Zhejiang Wanli University, 8 Qianhu South Road, Ningbo, Zhejiang, China; ^3^Ningbo Wanli Counterpart Collaboration and Anti-Poverty Research Institute, Ningbo, Zhejiang, China

## Abstract

As the primary industry, agriculture is a prerequisite for human survival and a basic industry of the national economy. As a result, the growth of agriculture is vital for the nation's socioeconomic development. The construction of ecological civilization and the reform and innovation of farmers' digital entrepreneurial behavior in the region are intimately correlated with the agricultural eco-environmental quality. Therefore, it is crucial for us to improve control and maintenance of the agricultural eco-environment. A requirement for directing the sustainable growth of the agricultural economy is evaluating and identifying the quality of the regional eco-environment and the issues it faces. In view of this, the study employs Jiangsu Province as a research example, builds a comprehensive index evaluation system, and uses the modified BP neural network to evaluate the agricultural eco-environmental quality in the target area between 2010 and 2020. First, the evaluation system is constructed from four dimensions: ecological resource status, environmental pollution degree, eco-environmental protection efforts, and agricultural development level, and 14 influencing factors are then screened out as specific secondary evaluation indicators. Second, a GA-BP model will be applied to comprehensively assess the quality of the agricultural eco-environment in the province over the past 10 years. The comprehensive score of the province's agricultural eco-environmental quality was calculated, and the quality level was classified by this. Meanwhile, the indicators' scores were paired with an analysis of each contributing factor's degree of change. The findings indicate that from 2010 to 2020, Jiangsu Province's agricultural eco-environment demonstrated a favorable trend, a reasonably high-quality level, and a tendency of continuous improvement from bad to good. The results of each indicator measuring the quality of the agricultural environment fluctuated, but overall they showed an upward trend. Finally, in order to offer a reference for agricultural eco-environment control and protection and a good ecological environment for farmers' digital entrepreneurship in the near future, countermeasures and suggestions are proposed for the restoration of the agricultural eco-environment in Jiangsu Province referring to the results of the research and the problems already present in the area.

## 1. Introduction

Agriculture is the backbone of our national economy, and the growth of the agricultural sector is one of the central issues that must be addressed to ensure the nation's and society's continued healthy and sustainable development [1]. As a result of China's remarkable advances in science, technological capability, and economic might, the digital entrepreneurial behavior of China's farmers and the country's agricultural digital economy have recently experienced exceptional breakthroughs. However, the rapidly expanding agricultural economy and agricultural production activities have also had a significant negative impact on the environment. These activities have caused problems such as soil, water, and air pollution from industrial triple waste emissions, indiscriminate deforestation, and overconsumption of ecological resources, all of which have resulted in significant damage to the environment. [2] The basis and guarantee for human survival, the development of agricultural entrepreneurship, and the upkeep of public health is a healthy eco-environment that is in good condition. According to studies that are pertinent to the topic at hand, ecological and environmental problems will result in a continuing deterioration of the conditions for agricultural output and will have a negative impact on the expansion of the agricultural economy. On the other hand, the steady expansion of the agricultural economy will make it easier for the government to carry out its plans for the regulation and protection of the environment [3]. Therefore, the development of an agricultural economy that is sustainable is inextricably linked to the maintenance of a healthy agricultural eco-environment. We will only be able to fundamentally achieve the coordinated development of economy and ecosystem, solve eco-environmental problems in economic and social development, and ultimately promote the digital entrepreneurial behavior of farmers and the construction of ecological civilization if we strengthen environmental control and maintenance in agriculture and strictly prevent the overexploitation of natural resources.

Because it is both a necessary condition and an essential guarantee for agricultural production, the standard of the eco-environment in which agriculture is practiced has a direct bearing on the expansion of the agricultural sector of the regional economy. The evaluation of the quality of the agricultural eco-environment has therefore become more and more important in order to prevent the deterioration of the agricultural eco-environment and to prevent problems before they occur. The establishment of a robust agricultural eco-environment not only fosters the growth of agriculture but also serves as an essential foundation for the achievement of sustainable regional development [4]. As can be seen, an all-encompassing analysis and forecast of the quality of the eco-environment surrounding agricultural production can help us gain an objective and in-depth understanding of the shifts and developments occurring in the agricultural eco-environment. This not only helps to control and conserve the ecological environment in the region, but also makes it possible to make better use of the resources that the environment provides. In order to provide a basic basis for environmental control and environmental construction [5], the evaluation of agricultural eco-environmental quality takes into primary consideration the information on agricultural ecological system attributes. Subsequently, in accordance with the chosen index system, the scientific evaluation method is utilized in order to evaluate the benefits and drawbacks of the agricultural eco-environment in a particular region. [6] This is done in order to fulfill the purpose of providing a foundation for environmental control and environmental construction. In the meantime, this is typically done from a systematic point of view, and the indicators are chosen in accordance with the conceptual framework of “pressure-state-response” [6]. The evaluation method, which functions as an important instrument, is another component that is essential for the accomplishment of a fruitful assessment of the ecological quality of agricultural land. At the moment, a great deal of theoretical frameworks is available for these evaluation methods. Among these are the fuzzy integrated evaluation model [7], the comprehensive index evaluation method [8], the hierarchical analysis method [9], the Grey relational analysis method [10], the principal component analysis method [11], and the artificial neural network method [12]. To construct an evaluation index system of agricultural eco-environmental quality for the study of sustainable development of an agro-ecosystem, literature [13–15] and others have used a combination of hierarchical analysis, the Delphi method, a multilevel fuzzy evaluation model, and other methods.

Within the Yangtze River, Economic Belt can be found in Jiangsu Province, which is characterized by its typical eco-environment and a medium to high level of agricultural growth. Jiangsu province was selected as the study area in order to facilitate the carrying out of an in-depth evaluation study on the ecological surroundings of agricultural operations. The evaluation method that is going to be used in this study is going to be a BP neural network technology that has been optimized by a genetic algorithm. This will allow for a comprehensive analysis of the factors that are having an effect on the quality levels of the agricultural eco-environment in this province. The relevant factors that have an impact on the quality of the agricultural eco-environment in our country are studied from an empirical perspective to provide appropriate theoretical support for the evaluation of agricultural eco-environmental quality in our country. Their weights are sorted and graded, and the degree of change of each influencing factor is analyzed. This is done to provide appropriate theoretical support for the evaluation of agricultural eco-environmental quality in our country. The following are the primary components of this research: building the evaluation index system should be the first step. We developed an evaluation index system for the agricultural eco-environment by studying the influencing factors, using the four primary evaluation indicators (ecological resources status, environmental pollution degree, eco-environmental protection efforts, and agricultural development level), and 14 influencing factors as specific secondary evaluation indicators. The primary evaluation indicators are: ecological resources status, environmental pollution degree, eco-environmental protection efforts, and agricultural development level. Second, in order to increase the evaluation model's objectivity as well as its level of intelligence, a BP neural network model that is based on a genetic algorithm has been developed as an evaluation method. In conclusion, based on the findings of the evaluation and the problems that already exist, suggestions and countermeasures are proposed for the purpose of restoring the agricultural eco-environment in Jiangsu Province in order to provide decision support for the development of agricultural ecological civilization. The use of a BP neural network as a method for evaluating the quality of the eco-environment is novel to this study, in contrast to other studies that have been conducted. This has the advantage of enabling the BP neural network to automatically calculate the weights of each indicator through the process of model training. As a result, problems associated with artificially determining weights and semi-qualitative in earlier evaluation methods are eliminated, and the reliability, objectivity, and comparability of evaluation results are enhanced.

## 2. Data and Methodology

### 2.1. Overview of the Study Area

Jiangsu plays an important part in the economy of the Yangtze River Delta region. It is located in the middle of the eastern coastal region of the Chinese mainland, and its borders are formed by the provinces of Shanghai, Zhejiang, Anhui, and Shandong. Its latitude ranges from 30°45′ to 35°20′ north, and its longitude ranges from 116°18′ to 121°57′ east. In addition to sharing a boundary with the Yellow Sea to the east, the Yangtze River, and the Huaihe River, the terrain of Jiangsu is primarily flat and contains a large number of lakes. Jiangsu Province is geographically located between the north and the south of China; as a result, the province's climate and vegetation exhibit characteristics of both the south and the north. Jiangsu experiences temperatures that range from 13.6 to 16.1 degrees Celsius on an annual basis, with the temperature trending downward from south to north. It receives between 704 and 1250 millimeters of precipitation annually, and the amount of precipitation that falls along the coast and in coastal areas is disproportionately higher compared to the amount that falls inland. Jiangsu has abundant rainfall, with little difference between north and south and a little variation between annual seasons. This is in comparison to other regions with the same latitude. As a result, Jiangsu enjoys the benefits of a pleasant climate, average annual precipitation, and excellent natural conditions for agriculture. This region is known for its high agricultural yields and serves as a significant hub for agricultural digital entrepreneurship in our nation.

Recently, with the substantial adjustment of the agricultural industry structure, the agricultural ecosystem in Jiangsu Province has undergone remarkable changes. With economic development, agricultural irrigation facilities, agricultural mechanization levels, and other agricultural production conditions have improved significantly, the structure and function of agricultural ecosystems have changed significantly, and agricultural production capacity has steadily increased. Meanwhile, the process of urbanization in rural areas has led to a sharp decrease in the area of arable land and serious damage and pollution of the eco-environment, and the conflict between the eco-environment, agricultural production, and social and economic development has become more and more acute. In light of this, the research choose Jiangsu Province as the target area to evaluate the quality of the agricultural eco-environment, which can provide scientific reference for the construction of agricultural ecology in the developed eastern regions of China.

### 2.2. Data Source and Processing

The data of the indicators in this study were obtained from Jiangsu Statistical Yearbook (2010–2020), China Environmental Yearbook (2010–2020), the ecological and environmental status bulletin of Jiangsu Province in the past years, and Easy Professional Superior (EPS) data platform.

In addition, this study standardized the original data on the basis of the established indicator system in combination with the uniqueness and actual condition of its own data, i.e., the indicators were divided into positive indicators and negative indicators. Based on the purpose of ensuring the accuracy of the analysis results, the above two types of indicators need to be processed as follows, and the calculation process is illustrated in formulas (1) and (2), respectively.

(1) $$\begin{array}{c} S_{ij}=\frac{o_{ij}-\min\left(o_{ij}\right)}{\max\left(o_{ij}\right)-\min\left(o_{ij}\right)}, \end{array}$$

(2) $$\begin{array}{c} S_{ij}=\frac{\max\left(o_{ij}\right)-o_{ij}}{\max\left(o_{ij}\right)-\min\left(o_{ij}\right)}, \end{array}$$

where *S*_*ij*_ denotes the index value after the standardization of *o*_*ij*_ and *o*_*ij*_ is the *j*th indicator value for year *i.*

### 2.3. Evaluation Index System

Agriculture's eco-environment is a complex system comprised of nature, biology, social economics, and technology, and it is influenced by both the natural environment and human activities [16]. As a result, its evaluation index system should be comprehensive and aligned with the goal of sustainable development, allowing the evaluation goal and the evaluation index to be organically linked to form a well-defined whole. This will make the evaluation goal and evaluation index more understandable. It can reflect global, long-term, local, current, and individual characteristics. It may also reflect comprehensive, current, and personal characteristics.

As a result, this study creates an evaluation index system for regional agricultural eco-environmental quality based on the principles of scientificity, availability, independence, and dynamics. This is accomplished through the use of pertinent literature. To begin, there are three layers in the evaluation system: the target layer, the criterion layer, and the index layer. The widely used pressure-state-response (PSR) system serves as a guide for the evaluation process [17]. A multi-level evaluation index system was built from four aspects using the aforementioned index construction principles, as shown in Figure 1.

As shown in Figure 1, the evaluation index system for the quality of agricultural eco-environments is composed of three layers. These layers are designated as the target layer, the criterion layer, and the index layer respectively. The target layer's primary function is to provide a description of the local agricultural eco-environment system's overall state as well as the dynamic changes that are occurring within it. The criterion layer's primary functions are to characterize the factors that constrain and affect the agricultural eco-environment system and to evaluate the variations that exist within the ecosystem. These are the two primary areas of focus for the criterion layer. It consists primarily of these areas: ecological resource status is a method that is used to reflect the condition of the natural environment in the surrounding area. The level of environmental pollution describes the degree to which farmland, water bodies, and the atmosphere in the target area are polluted with harmful substances. The efforts of eco-environmental protection, which is a reflection of all of the efforts made to safeguard the ecological balance of agriculture, minimize the use of natural resources, and prevent pollution. Agricultural development level reflects the ability of the target region to generate and maintain a particular annual growth rate of GDP. The indicator layer, which is a directly measurable indicator that describes the relevant element of the criterion layer [18], is the most fundamental component of the indicator system. In this particular investigation, the indicator layer is made up of a total of fourteen different environmental factors.

### 2.4. Research Methodology

Determining the weights of the indicators in the evaluation system is a critical component of assessing agricultural eco-environmental quality. However, as previously stated, human factors easily disrupt traditional evaluation methods, resulting in a lack of objectivity and scientificity in evaluation results. As a result, the BP algorithm was further optimized with the genetic algorithm in this study, and the optimized GA-BP algorithm was used as the evaluation method to determine the weights of each indicator [19]. In this way, not only can the self-learning and self-adaptive advantages of the BP neural network be used, but also the better global search ability of the genetic algorithm, greatly improving the scientific and accurate results of model evaluation.

Backpropagation (BP) neural networks are also referred to as multilayer feedforward neural networks. It is, in other words, a multilayer feedforward network that has been trained by an error-based backpropagation algorithm. A typical BP network has a three-layer network structure with an input layer, a hidden layer, and an output layer, as shown in Figure 2.

It is clear from looking at Figure 2 that the learning process of the BP neural network is primarily comprised of two parts: A portion of the total is made up of forwarding propagation. That is, in the case of the input sample data, it is first subjected to processing and calculation with the help of the input layer and the hidden layer, and then the output layer generates the results. The other part of this process is called backward propagation. The weights and biases of each layer of the network are sequentially adjusted until the model converges. These adjustments are made in accordance with the error that exists between the actual value produced and the expected value. In recent years, the use of the BP neural network has become increasingly popular among academics as a result of the distinct advantages it offers when dealing with nonlinear data. On the other hand, as the range of applications grows incrementally, the limitations of the technology, such as the need for local miniaturization and a slow convergence speed, are coming into sharper focus.

As a solution to the problems outlined above, the researchers decided to use a novel GA-BP neural network model for their investigation. This model was created by fusing a genetic algorithm [20] with BP neural network. In this particular representation, the initial weights of the BP neural network are optimized with the help of a genetic algorithm. After that, the BP neural network is trained using the initial weight that was just determined as its initial weight. The performance of the trained network model is then evaluated, as the last step.

It is also essential to keep in mind that the evaluation performance of BP neural networks can be significantly impacted by the quality of the connection weights. This is something that must be kept in mind at all times. As a consequence of this, the conventional method for determining the connection weights of the network is to compute the sum of the squared errors. Formulas illustrate the steps of the calculation process (3).

(3) $$\begin{array}{c} E=\sum_{M}\sum_{N}\left(P_{N}-S_{N}\right), \end{array}$$

where *S*_*N*_ represents the input signal, *P*_*N*_ is the predicted value, and *M* and *N* denote the number of samples and the number of nodes in the output layer, respectively. The training process of the GA-BP neural network model is illustrated in Figure 3.

After that, the trained GA-BP network model was utilized in order to finish the comprehensive evaluation of the eco-environmental quality of agricultural practices. However, in order to conduct a more intuitive evaluation of the agricultural eco-environmental quality, we also conducted a graded evaluation of the agricultural eco-environmental quality, with reference to the comprehensive evaluation scores calculated by the GA-BP network model. This allowed us to evaluate the agricultural eco-environmental quality in a more nuanced manner.  Figure 4 provides a visual representation of the specific classification results.

According to the level, the quality of the agricultural eco-environment was rated as “excellent,” “good,” “medium,” “poor,” and “bad,” as shown in Figure 4. These grades were assigned based on the level going from high to low. A higher total score on the evaluation indicates a higher level of ecological and environmental quality in agricultural practices. On the other hand, if the level of ecological and environmental quality in agricultural production is lower.

Last but not least, the findings of the aforementioned research led to the application of the GA-BP network model to the assessment of the eco-environmental quality of agricultural land, and the operation process in its entirety is depicted in Figure 5.

## 3. Results and Analysis

According to the above research method, the raw data of each indicator layer were brought into the GA-BP model to determine the weights of each indicator of Jiangsu agricultural eco-environmental quality from 2010–2021. The results as illustrated in Table 1.

From the weights of each indicator in Table 1, we can see that the ecological resource status has the greatest influence on the quality of the agricultural eco-environment, reaching 0.426, while the weights of its two second-level indicators, effective irrigation area, and water area rate are both larger than 0.1, especially the former with a weight of 0.189. The second is the degree of environmental pollution, with a weight of 0.248, and the weight of pesticide use intensity in its secondary indicators is also the largest, exceeding 0.1. The third is the level of agricultural development, with a weight of 0.217. The weights of its secondary indicators are more evenly distributed, hovering around 0.7. The least influential is the efforts of eco-environmental protection, with a weight of only 0.162. Among them, the weight of the nature reserve area in its second-level evaluation index is the smallest, only 0.031.

According to the above weighting results, the comprehensive score of agricultural eco-environmental quality of Jiangsu Province from 2010 to 2020 is obtained, and then its grade in all years will be obtained according to the grade classification criteria (as displayed in Figure 3). The corresponding results are illustrated in Table 2.

As shown in Table 2, the level of agricultural eco-environment quality in Jiangsu Province generally shows an increasing trend year by year. However, in terms of the overall score and ranking, there is a certain degree of volatility on the whole. For example, although the environmental quality levels in the two years (2016 and 2017) are the same, the comprehensive score of eco-environmental quality in 2017 has decreased. In addition, the comprehensive scores in 2014 and 2016 both increased by more than 0.1, showing a large increase. In terms of quality grades, the eco-environmental quality grade of Jiangsu Province gradually transitions from bad to good. 2010 is bad, 2011–2012 is poor, 2013–2015 is medium, and 2016–2020 is good. Therefore, it can be concluded that the level of agricultural eco-environmental quality in Jiangsu Province is improving continuously.

In order to understand the specific impact of each indicator on the quality of Jiangsu's agricultural eco-environment, the comprehensive score was divided into the scores of each first-level indicator. According to the indicator scores, the degree of change of each influencing factor in 2010–2020 is specifically analyzed from different levels. The detailed results are shown in Figure 6.

As can be seen from Figure 6, the scores of the second-level indicators of agricultural eco-environmental quality in Jiangsu province are generally fluctuating during the period of 2010–2020. The score of the ecological resource status fluctuate the most in 2014, 2017, and 2020, indicating that the ecological resource situation in Jiangsu province is generally the best in these years. The ecological resources of the province generally showed a decreasing trend from 2011 to 2013, and the lowest score was in 2013. The ecological resource situation in 2014–2020 showed an overall upward trend, but it declined in 2018. The score of environmental pollution fluctuates widely, with the highest score in 2018 and the lowest score in 2010. Roughly speaking, it has a volatile uptrend. The lowest score of environmental protection is in 2012, and the highest is in 2020. The scores of this indicator in other years are not much different, with small fluctuations. However, in the past three years, the overall score of this indicator has shown a trend of continuous improvement. It can be concluded that people have been paying more and more attention to environmental protection in recent years. During the period 2010–2020, the scores of agricultural development indicators have generally increased year by year. As a whole, agricultural development has an upward trend. This shows that Jiangsu Province attaches importance to the development of agriculture, and there is a significant improvement in both economic production and technology levels. In summary, since the scores of the four indicators of ecological resources, environmental pollution, environmental protection, and agricultural development have an overall increasing trend, the comprehensive indicator scores will also have an increasing trend. This is consistent with the conclusion of the previous comprehensive score analysis.

## 4. Discussion and Suggestions

### 4.1. Discussion

The quality of Jiangsu's agricultural eco-environment was evaluated in this study using the GA-BP model at four different levels: ecological resource status, environmental pollution degree, eco-environmental protection efforts, and agricultural development level. Based on the findings of the aforementioned thorough evaluation, a summary of Jiangsu Province's agricultural eco-environment growth from 2010 to 2020 is provided. Even though Jiangsu Province has made significant progress in agricultural eco-environment control. It should not be overlooked that there are still some problems in the construction of the agricultural eco-environment at present. It mainly includes the following points:

1. The overall level of agricultural eco-environmental quality is not high. During 2010–2020, the agricultural eco-environmental quality of Jiangsu Province exhibits a development trend from bad to good, but the overall level is not high. Although after nearly 10 years of unremitting efforts, the overall environmental quality score in 2020 exceeds 0.8, it still does not reach the level of excellence, and the agricultural eco-environment control needs to be further strengthened.
2. The improvement of the agricultural eco-environment is not obvious. Looking at the changing trend of the agricultural eco-environmental quality in Jiangsu Province from 2010 to 2020, it can be found that since 2016, the agricultural eco-environmental quality of the province has been stable for a long time at a “good” level. The upward trend and improvement effect are not significant.
3. The irrational use of ecological resources has restricted the improvement of the quality of the agricultural eco-environment. Jiangsu Province has a unique geographical advantage, abundant light and rainfall, and relatively abundant natural resources. However, these ecological resources are restricted by external natural factors and cannot be changed in the short term. In the evaluation system of agricultural eco-environmental quality, the indicator plays a decisive role in the evaluation results, thus greatly limiting the improvement of agricultural eco-environmental quality.
4. The degree of pollution and damage is relatively severe, and the burden on the ecosystem is significant. The economic development level of Jiangsu Province is far ahead of China and belongs to the economically developed region. But since science, technology, and society have advanced so quickly, environmental pollution from industrial production has also emerged and gotten worse. The environmental pollution level indicator's overall score is much lower than the scores for the other three indicators from 2010 to 2020. The original data, particularly the evaluation scores of the two secondary indicators of “fertilizer application intensity” and “pesticide application intensity,” indicate that there are significant issues. The quality of the agricultural ecological environment is gravely threatened by the province's continued comparatively high levels of environmental pollution and destruction.
5. Insufficient efforts in agricultural eco-environmental protection. It is evident from the evaluation of environmental protection efforts that, between 2010 and 2015, the target area's overall nature protection degree showed a steady rising trend and that the environmental protection effort gradually rose. However, during the period from 2016 to 2020, the environmental protection efforts have increased compared with the previous years. The environmental protection efforts in 2017 and 2018 decreased compared with 2016 and continued to decrease after a brief rebound. Therefore, the agricultural eco-environmental protection is not strong enough, resulting in the agricultural eco-environment is not effectively and continuously protected.

### 4.2. Suggestions

A good quality of agricultural eco-environment is an indispensable part of ensuring sustainable development of the agricultural economy. Jiangsu has abundant agricultural resources and is important to the development of China's agriculture. To improve the economic environment and encourage the construction of the Yangtze River Economic Belt, it is crucial to address the problems with the region's agricultural eco-environment and utilize the agricultural resources efficiently. To this end, in response to the previous analysis of the comprehensive evaluation of the quality of the agricultural eco-environment in Jiangsu Province and the main problems existing in the agricultural eco-environment of the province at present, the following suggestions are made in a targeted manner.

1. Optimize the governance system of the regional agricultural eco-environment and do a top-level design. With the purpose of improving the overall level of Jiangsu's agricultural eco-environment, we should first optimize the governance system of the regional agricultural eco-environment and strengthen top-level design. First, we must remain problem-oriented, integrate the development characteristics of the agricultural eco-environment of the target region, and conduct a scientific, comprehensive, reasonable, and balanced top-level design. Second, we should adhere to the concept of sustainable development, proceed from the overall situation, and formulate regional agricultural eco-environment governance strategies according to local conditions. Thereby narrowing the differences between various regions in the province, promoting balanced development, and improving the overall level of agricultural eco-environment in the region.
2. Give full play to the utility of the soft environment and establish a pluralistic governance mechanism. In addition to paying attention to the hardware requirements needed to restore the agricultural eco-environment, we need also pay attention to the usefulness of the external soft environment in order to strengthen the improvement effect of the agricultural eco-environment. To increase the efficiency of environmental governance, it is first important to fully exploit the function of the external soft environment, which includes policies, culture, ideologies, and protective consciousness. Second, focus on maintaining a good human environment for the agricultural eco-environment, and increase the attention and investment in the soft environment of agricultural ecology. Finally, enhance the participation of farmers, widely adopt their opinions and suggestions on the construction of agricultural eco-environment, and raise their awareness on the protection of agricultural eco-environment.
3. Combination of treatment and prevention to improve the environment and lessen the impact of natural disasters on agriculture. The harm caused by natural disasters is a significant factor that prevents the agricultural eco-environment from improving. Natural disasters are readily ignored since they are unavoidable. Natural disasters are incredibly destructive, common, and unexpected, frequently resulting in concentrated and catastrophic damage to crops and seriously threatening agroecological health. In order to lessen the harm that natural disasters cause to the agricultural eco-environment, we should concentrate on prevention, increase the building of agricultural infrastructure, and take multiple measures. Second, in order to build a healthy natural eco-environment, we should encourage the restoration of the agricultural eco-environment and do a good job of treating and restoring farmland that has been damaged by disasters or industrial pollution.
4. Strengthen agricultural scientific and technological innovation, and rationalize the use of agricultural ecological resources. On the one hand, encourage the development and use of agricultural science and technology in accordance with regional conditions. Following the principles of green production, energy conservation, and efficiency, new species of animals and plants are chosen, and the level of agricultural mechanization is vigorously increased, all of which contribute to the sustainable development of agricultural ecology and agricultural economy. On the other hand, accelerate the exploration, innovation, and pilot application of key and core technologies for ecological and environmental protection governance. For instance, encouraging the recycling of straws to prevent environmental pollution from incineration. Application of chemical amendments to boost the soil's ability to purify itself, rational fertilization, and prudent farming scheduling all help to encourage the development of a sustainable agriculture industry.
5. Increase environmental protection efforts and strengthen environmental control and regulatory mechanisms. First, local governments should increase environmental protection efforts, invest more special funds to reduce urban wastewater and waste gas emissions, strengthen arable forest protection and quality construction, focus on agricultural ecological restoration, and return a healthy and safe agricultural eco-environment to the region. Second, we should raise awareness of agricultural eco-environmental protection, cultivate new professional farmers with modern agricultural production skills, and promote the transformation of the traditional crude agricultural production model to a modern digital entrepreneurship model to ensure that the agricultural economy follows a sustainable development path. Finally, establish a strict environmental control and supervision mechanism. In accordance with the principle of “local management, comprehensive coverage, graded responsibility, responsibility to the person, dynamic management,” the grid management of environmental control is fully implemented.

## 5. Conclusions

The quality of the eco-environment in agricultural settings is an essential component in the process of ensuring the agricultural economy will continue to grow sustainably. The extent to which human activities are having an impact on the quality of the agricultural eco-environment can be revealed and predicted by conducting an assessment of the quality of the agricultural eco-environment. This helps to provide a reference basis for the formulation of agricultural environmental planning, agricultural environmental zoning, and agricultural regulations, in addition to providing a basis for environmental control and digital entrepreneurship among farmers. As a consequence of this, Jiangsu Province is selected as the focus of the research, and a BP neural network model that is derived from genetic algorithms is used to evaluate the quality of the agricultural eco-environment in Jiangsu Province from the years 2010 to 2020. According to the findings of the evaluation, the agricultural eco-environmental quality in Jiangsu Province has gradually improved over the past 10 years, and the quality level has been optimized in the direction of bad, poor, medium, and good over that time period as well. The level of environmental pollution and agricultural development have the greatest influence on the quality of the agricultural eco-environment, followed by the ecological resources, which have the greatest influence on the quality of the agricultural eco-environment; and in the evaluation system for the quality of the agricultural environment, the eco-environmental protection efforts have the least influence. In addition, the results of these four first-level indicators are currently exhibiting a state of fluctuation, even though the overall trend is upward. In light of the problems that were discovered in the aforementioned study, some preventative actions and recommendations for agricultural eco-environmental control and restoration in Jiangsu Province are presented in the conclusion of this article.

Modern agriculture is currently moving in the direction of creating ecological agriculture that is high-yielding, of high quality, and highly efficient in order to achieve a high degree of unity and the sustainable development of economic, social, and ecological benefits. This is being done in order to pursue a high degree of unity and the sustainable development of economic, social, and ecological benefits. This is done to maintain a healthy eco-environment for agricultural production. As a consequence of this, the evaluation system that was developed during the course of this study has the potential to not only assess the current state of the agricultural eco-environment in China but also act as a reference point for decisions regarding the development of ecological agriculture. In addition to this, it seeks out innovative methods to investigate the digital entrepreneurial behavior of farmers. However, it is important to emphasize that although the 14 second-level indicators [20] and four first-level indicators that we chose to include in the evaluation system that we built for this study are very relevant to the agricultural eco-environment and are somewhat typical, they are not exhaustive enough to serve as the sole basis for the evaluation. In order to get the most accurate findings out of the research being done, the choice of indicators being used needs to be refined as the project moves forward. In addition to this, there is a requirement for a more in-depth comparison of samples gathered from different eras.

## Figures and Tables

**Figure 1:** Agricultural eco-environment evaluation index system.

**Figure 2:** BP neural network structure.

**Figure 3:** Training process of GA-BP network model.

**Figure 4:** Grade classification.

**Figure 5:** Application of GA-BP network model in the evaluation of agricultural eco-environmental quality.

**Figure 6:** Distribution of scores for each indicator from 2010 to 2020.

**Table 1:** The weights of each indicator of agricultural eco-environmental quality.

Criteria layer (first-level indicator)	Weights of first-level indicators	Index layer (second-level indicator)	Weights of second-level indicators
Ecological resource status	0.426	Per capita arable land	0.062
		Effective irrigation area	0.189
		Forest cover rate	0.042
		Water area rate	0.117

Environmental pollution degree	0.248	Pesticide use intensity	0.107
		Fertilizer use intensity	0.087
		Disaster area rate	0.048

Eco-environmental protection efforts	0.162	Investment in environmental governance	0.063
		Area of nature reserve	0.031
		Sewage treatment rate	0.068

Agricultural development level	0.217	Per capita disposable income of farmers	0.032
		Gross agricultural output	0.072
		Grain yield per acre	0.063
		Agricultural mechanization rate	0.067

**Table 2:** Comprehensive scores, quality grades, and rankings.

Year	Survey item		
	Score	Grade	Ranking

2010	0.334	Bad	11
2011	0.361	Poor	10
2012	0.382	Poor	9
2013	0.528	Medium	8
2014	0.634	Medium	7
2015	0.671	Medium	6
2016	0.782	Good	4
2017	0.763	Good	5
2018	0.784	Good	3
2019	0.792	Good	2
2020	0.826	Good	1

## Data Availability

The labeled dataset used to support the findings of this study are available from the corresponding author upon request.
